The article "Novel Prediction Model for COVID-19 in Saudi Arabia Based on an LSTM Algorithm" was retracted in 2023. Reasons: signs of a paper mill; compromised peer review; unreliable results or conclusions.

# Novel Prediction Model for COVID-19 in Saudi Arabia Based on an LSTM Algorithm

**DOI:** 10.1155/2021/6089677

**Published:** 2021-12-18

**Authors:** Eman H. Alkhammash, Haneen Algethami, Reem Alshahrani

**Affiliations:** Department of Computer Science, College of Computers and Information Technology, Taif University, P.O. Box 11099, Taif 21944, Saudi Arabia

## Abstract

The rapid emergence of the novel SARS-CoV-2 poses a challenge and has attracted worldwide attention. Artificial intelligence (AI) can be used to combat this pandemic and control the spread of the virus. In particular, deep learning-based time-series techniques are used to predict worldwide COVID-19 cases for short-term and medium-term dependencies using adaptive learning. This study aimed to predict daily COVID-19 cases and investigate the critical factors that increase the transmission rate of this outbreak by examining different influential factors. Furthermore, the study analyzed the effectiveness of COVID-19 prevention measures. A fully connected deep neural network, long short-term memory (LSTM), and transformer model were used as the AI models for the prediction of new COVID-19 cases. Initially, data preprocessing and feature extraction were performed using COVID-19 datasets from Saudi Arabia. The performance metrics for all models were computed, and the results were subjected to comparative analysis to detect the most reliable model. Additionally, statistical hypothesis analysis and correlation analysis were performed on the COVID-19 datasets by including features such as daily mobility, total cases, people fully vaccinated per hundred, weekly hospital admissions per million, intensive care unit patients, and new deaths per million. The results show that the LSTM algorithm had the highest accuracy of all the algorithms and an error of less than 2%. The findings of this study contribute to our understanding of COVID-19 containment. This study also provides insights into the prevention of future outbreaks.

## 1. Introduction

Emerging and reemerging viruses pose severe challenges to public health. Coronaviruses are a family of highly pathogenic enveloped RNA viruses, which are widely transmitted among humans [1]. In late December 2019, a new coronavirus pandemic erupted unexpectedly in Wuhan, China, posing a serious threat to everyday human life. The new virus, dubbed severe acute respiratory syndrome coronavirus 2 (SARS-CoV-2) by the World Health Organization [2], causes coronavirus disease (COVID-19), which often results in death [1]. During the weeks that followed, the virus broke out in China and quickly spread to other countries, causing global panic. As of late February 2020, at least 38 countries had reported 83,652 confirmed cases [2], demonstrating the pathogen's astounding propagation speed [3].

To combat the pandemic, many countries have implemented protective measures, such as mandatory quarantines or even massive closures. The pattern of the outbreak's spread and speed varies from country to country [4]. The rate of spread within a country is specifically determined by factors such as weather conditions, city population density, level of urbanization, social cohesiveness, and cultural factors that can be identified as influential factors of human-to-human transmission of the virus. Thus, to fully control the epidemic, effective protective measures must be tailored to each nation's environment, social factors, and culture.

The variable transmission of SARS-CoV-2 raises the question “what are the factors influencing the spread of the virus in Saudi Arabia?” Saudi Arabia was one of the first countries to react and demonstrated innovative leadership characteristics when dealing with COVID-19.  Figure 1 shows the status of COVID-19 in Saudi Arabia as of May 7, 2020. The Saudi government has developed multifaceted public health interventions, such as home quarantine, nationwide lockdowns, traffic and travel bans, and centralized isolation of infected people. The quarantine of symptomatic individuals, close contacts of infected individuals, and travelers from other countries were among the measures taken by the government to slow the spread of the virus. Additionally, the country's Ministry of Health [5] provided early treatment for infected people to prevent further complications. This was established by selecting 25 hospitals, with up to 80,000 hospital beds, 2,200 of which were for isolating suspected/quarantined cases and 8,000 intensive care unit (ICU) beds for treating COVID-19 patients [6]. These interventions, in conjunction with universal symptom screening, substantially slowed the transmission rate [5].

The pandemic has a negative influence on the economic and social aspects of society. Many manufacturers are working on COVID-19 vaccines, which aim to minimize health damage and reduce the chances of viral mutation [7]. To combat the pandemic and slow its spread, there is a pressing need to develop effective models to identify the factors that could increase the number of infected people. The current global COVID-19 situation clearly indicates that new diseases and illnesses may emerge rapidly. Understanding the factors that contribute to the spread of these viruses is essential to slow their spread and prevent infections. Moreover, knowing the spread rate of a disease is essential for managing healthcare services provided to those affected by it. Therefore, there is a need to develop tools and algorithms that can effectively address outbreaks and pandemics as new viruses emerge.

Neural network (NN)-based prediction models have the potential to make highly accurate predictions. NNs open up new possibilities in epidemiology. The merit of our study is that we compared the performance of different models for prediction analysis of COVID-19 cases: a fully connected NN, long short-term memory (LSTM), and transformer model (TM). They were used to predict essential factors, such as the number of cases, deaths, vaccinated, extreme poverty, handwashing facilities, weekly hospital admissions, weekly hospital admissions per million, ICU patients per million, weekly ICU admissions per million, weekly ICU admissions, hospital patients per million, hospital patients, ICU patients, new vaccinations, total vaccinations per hundred vaccinations, new vaccinations smoothed per million, new vaccinations smoothed, new deaths per million, and the extent to which people adhered to government regulations during quarantine.

Most epidemics, including COVID-19, exhibit distinct patterns of spread. The disease does not manifest in the same way in every country or region of a country [4]. In some cultures, families socialize more often, whereas in others, they prefer a more solitary lifestyle. Moreover, different population densities in cities or the reliance on public transportation can influence the transmission rate. If it is assumed that the virus behaves consistently worldwide, the prediction results may be inaccurate. Understanding the speed and spread of the virus at the local and national levels is critical for developing the best models possible, which motivated us to use three different models to examine and compare influential factors in Saudi Arabia.  Figure 2 shows the spread of COVID-19 in different cities in Saudi Arabia.

Modeling aids in identifying potential determinants of COVID-19 spread and in determining the areas and populations that are most vulnerable. The goal is to effectively identify COVID-19 spread factors and to evaluate and validate the accuracy of the developed model.

## 2. Related Work

Some researchers have focused on using statistical analysis to understand the spread of COVID-19. In [3], basic statistics and linear regression were used to investigate the daily transmission dynamics of the virus in infected countries while evaluating the effectiveness of control measures. In [8], simple statistical methods were used to examine the correlation between disease severity and environmental, economic, and social factors. Statistics-based research findings are limited to understanding the current state of the outbreak.

In [9], a stochastic model was developed to calculate the probability of transmitting the virus from one area to another. This study was based on the traffic between these areas in China. Although the model could predict virus propagation, it considered only travel as a factor. The authors of [10] studied the effect of meteorological parameters such as temperature and relative humidity in China from January 20, 2020, to February 29, 2020. The study found a positive association between deaths and diurnal temperature range and a negative association between deaths and relative humidity.

Another study investigated the correlation between the weather and spread of COVID-19 in Jakarta [11]; the study included several weather factors: minimum, maximum, and average temperatures, humidity, and the amount of rainfall. The Spearman-rank correlation test was used, and it was concluded that the average temperature had a significant influence on the spread of COVID-19. Another study [12] conducted in 21 countries showed that high temperatures influence COVID-19 spread and reduce initial contagion rates.

Many studies indicate that artificial intelligence and deep learning models have highly accurate predictions for specific occurrences [13, 14]. Recently, both machine learning and deep learning techniques have been used for time-series forecasting and have produced excellent results. Several deep learning models with remarkable results were used to predict new COVID-19 cases, the rate of change, and other factors.

NNs can precisely predict the behavior of a pandemic. The authors in [15] proposed an approach based on binary classification and regression analysis considering daily weather parameters such as wind, temperature, humidity, and the city's density. The study was conducted in Hubei province in China and concluded that humidity and temperature significantly impact confirmed cases. An average relative humidity of 77.9% positively affected the confirmed cases, whereas an average temperature of 15.4°C negatively affected the confirmed cases.

Another study linked COVID-19 propagation to economic conditions in China. The study used data science and machine learning algorithms to explain key factors in the spread of the virus [16]. The authors of [17] investigated the relationship between the spread of epidemics and increased transportation and trade. The study aided in understanding how economic conditions are linked to disease spread.

The authors of [18] used NNs to predict risk categories per country using Bayesian optimization along with the trend and weather data. The fuzzy rule was used to classify a country's risk level (high, medium, and recovering). The average accuracy of the proposed model was 78% for 170 countries.

Another study proposed a COVID-19 forecasting model based on improving the flower pollination algorithm and combining it with the salp swarm algorithm [19]. The proposed model was tested on confirmed cases in the USA and China, where it was found to be promising. The authors of [20] applied the autoregressive integrated moving average (ARIMA) to predict the prevalence of COVID-19 in Italy, Spain, and France during the period from February 21 to April 15, 2020. The ARIMA time-series model was useful in predicting the outbreak trend in the three countries, which can ultimately help authorities plan and manage the outbreak situation in the future.

Perc et al. [7] proposed an iteration method to forecast COVID-19 in various countries such as the USA, Slovenia, and Germany. The proposed approach was based on daily confirmed cases, expected recoveries, and deaths. The results showed that the spread of COVID-19 should be less than 5% each day to control the pandemic and attain a plateau. Furthermore, another study suggested that the number of cases and population intensify the spread of COVID-19 over time [21]. However, the rate of spread of COVID-19 tends to decrease in larger cities compared with smaller ones.

In another study, a hybrid deep NN based on computed tomography and X-rays for predicting COVID-19 was proposed. The datasets used in the study were collected from various sources, for example, GitHub, the COVID-19 Radiography Database, and Kaggle. The proposed algorithm achieved a classification accuracy of 99% on the test dataset [22]. Another approach, COVID Inception-ResNet model (CoVIRNet), was proposed to diagnose COVID-19 patients using chest X-rays [23]. This approach used a combination of deep learning and machine learning models and achieved an accuracy of more than 95% [23].

The authors of [24] provided a global and country-specific comparative analysis of time-series forecasting using ARIMA, LSTM, stack LSTM (SLSTM), and Prophet approaches. The analysis predicted the cumulative COVID-19 new cases. It also included different features of correlation to identify the best prediction model through statistical hypothesis testing. In terms of accuracy, SLSTM outperformed the other models. In statistical analysis, ARIMA outperformed the LSTM model. Overall, the SLSTM model performed better than the other models.

The authors of [25] compared six different prediction models, including ARIMA, nonlinear autoregressive NN, and LSTM, to predict the cumulative confirmed new cases and the total increase rate. The mean absolute percentage error values of the LSTM model showed better accuracy than those of the other models. Authors of [26] also used the LSTM model to estimate the number of confirmed cases and compare the growth rate. The model showed 92.67% accuracy.

Our work contributes to the existing literature threefold.

Our analysis is linked to the social and epidemiologic literature on factors and measures to prevent and control an outbreak.

Our study focuses on pandemic spread in Saudi Arabia and can be replicated to complement epidemiologic studies in countries with similar social and environmental aspects, such as Kuwait and Bahrain.

We introduce a comparative analysis of three different deep learning time-series prediction models for predicting COVID-19 cases for up to the subsequent five days.

The main factors are previous cases and the extent to which people adhere to government's regulations. In this study, we used a fully connected NN, LSTM, and TM. These models exploit historical data of confirmed cases, and their main difference is the number of days that they assume impact the estimation process.

## 3. Methodology

The proposed method consists of three main phases: (1) collection, preprocessing, and preparation of data on COVID-19 cases in Saudi cities; (2) identifying features and predictors; and (3) applying the three NN models to predict outcomes. The objective was to develop a predictive model for the probability of the spread of COVID-19 in a specific area of Saudi Arabia.  Figure 3 illustrates the block diagram used to build the predictive model for this study. The details of each phase are explained in the following sections.

The data collected are the input of the model. In this study, the daily data of COVID-19 cases in Makkah Province were selected with mobility data from Makkah Province as a case study. Both datasets were selected for the same period. Subsequently, each model was trained and tested individually using the data collected to build the model. In this study, three models, a fully connected deep NN (DNN), LSTM, and TM, were used separately. For all models, the construction stage was the same. We used 80% of the data for training and 20% for verification (i.e., the test dataset). This means that the finalized model can predict the outcomes of the cases in the test dataset. The prediction is the result of the estimation processes, where the performance of the model is compared with the predicted outcomes. The final result was the predicted future cases of COVID-19.

### 3.1. Data Collection and Preparation

The optimization of the model accuracy depends on the preprocessing of the selected data and model validation. Daily data of COVID-19 cases in Makkah Province were selected to predict the number of new cases from February 2020 to June 2021. Dates were selected based on the arrival date of COVID-19 in Saudi Arabia, which was March 2, 2020, after the first Saudi citizens tested positive for COVID-19. Consequently, the number of confirmed cases and deaths began to rise. Makkah Province was selected because it is the third largest and most populated province in Saudi Arabia. It accounts for 26.29% of the entire Saudi population. Hence, a large COVID-19 spread in this region can cause more damage than in any other region.  Figure 4 shows the total COVID-19 cases in Makkah Province from February 2020 to June 2021.

Twenty features were selected for this study. The features included people vaccinated, people fully vaccinated, people vaccinated per hundred, people fully vaccinated per hundred, extreme poverty, handwashing facilities, weekly hospital admissions, weekly hospital admissions per million, ICU patients per million, weekly ICU admissions per million, weekly ICU admissions, hospital patients per million, hospital patients, ICU patients, new vaccinations, total vaccinations per hundred, total vaccinations, new vaccinations smoothed per million, new vaccinations smoothed, new vaccinations smoothed, and new deaths per million. All these data were reported by the Ministry of Health in Saudi Arabia [5].

Several factors influence the spread of COVID-19 in Saudi Arabia and play a crucial role in increasing the risk of infection.  Figure 5 depicts the different demographics of COVID-19 confirmed cases in Saudi Arabia, where 92% of the cases were adults who are more likely to affect others owing to their mobility.

To limit the spread of COVID-19, the government has enforced guidelines, including self-quarantine, partial curfews, and limiting traveling in and out of Saudi Arabia, such as hajj and umrah at Makkah. Lockdowns were enforced between April 21 and May 11, between 6 pm and 6 am. However, during the pandemic peak, between May 23 and May 27, 24-hour curfews were enforced. Lockdowns included staying at home; only people going out to purchase supplies and essential workers with permits were allowed to go out. These policies have contributed to a reduction in the spread of COVID-19. Therefore, in this study, mobility data were used as predictors, that is, features. Data for the Makkah Province were obtained from Google COVID-19 Community Mobility Reports from February 2020 to June 2021. The report describes six movement trends: retail and recreation, groceries and pharmacies, parks, transit stations, workplaces, and residential areas [27]. These data were measured as percentage change from a baseline.  Figure 6 presents an example of the percentage change from baseline mobility data during the same period of COVID-19 cases.

The factors were used in the model as predictors, that is, features. Feature extraction was used in this study to manage missing values and handle nonnumeric values. The data sources used are presented in Table 1.

Missing values, duplicate columns, and columns with the same values were fixed or dropped during data preprocessing. The time column was used to join mobility data with daily COVID-19 case data to determine whether mobility data were compatible with dates for all periods of COVID-19 case data.

### 3.2. Feature Selection

The first step is to understand the distribution of the model and whether the information in the dataset has any correlation relationship. Model accuracy is optimized by preprocessing the selected data and model validation. Hence, this study aimed to validate the proposed data-driven model by identifying the main factors affecting the spread of COVID-19 in Saudi Arabia, based on the collected data.

To measure citizens' adherence to self-quarantine and government guidelines, we collected mobility data for Makkah Province from Google COVID-19 Community Mobility Reports. The reports plot movement trends geographically across different places, such as groceries and pharmacies, parks, workplaces, and residential areas [27]. These factors are used in the model as predictors, where the predictor encoding is used in the model by identifying their correlation.

### 3.3. Artificial Neural Network Predictive Models

To build a predictive model, patterns were identified in a group of data to obtain answers [28]. Prediction models using NN can achieve high accuracy and thus can be used to develop tools and algorithms that can effectively address outbreaks and pandemics as new viruses emerge, opening new possibilities in epidemiology.

The time-series forecast aims to predict a series of discrete data points equally spaced in time [29]. DNNs have been extensively used as time-series forecasters; for example, convolutional neural networks, LSTM [30], transformers, and fully connected DNNs [31] have been used for COVID-19 cases forecasting.

This study used three time-series NN models to predict the number of COVID-19 cases for up to five days. The input layer feeds predictors {*A*, *B*,…, *P*} as past data values into the hidden layer. Predictors included previous case information and the extent to which people adhered to government regulations, as described in Section 3.2. The hidden layer takes the predictors using mathematical functions that modify the input data. The output layer gathers predictions made in the hidden layer and produces a prediction. Hence, the predictive models cover the training, testing, and estimation processes.

A fully connected DNN is a feedforward network that contains fully connected layers. It is used because it does not require any assumptions about the input: it is a general application of an artificial neural network. Hence, it can be applied to different types of areas. Note that for *n* inputs and *m* outputs, the number of weights is *n* × *m* [32]. LSTM is a recurrent network architecture combined with a gradient-based learning algorithm [33]. One advantage of LSTM is its ability to learn even with noisy, incompressible input sequences without loss of efficiency. A transformer is a DNN model that deals with sequential input data points used in the input representation [31].

In this study, TM was based on the work by [34], with the attention mechanism described in [30]. This is because input is not necessarily handled in order. However, this mechanism provides a context for any location in the input data points. Furthermore, the training process occurred in parallel, which allows for training with larger datasets. Additionally, the group linear transformations (GLT block) were inspired by Zhuang et al. [34] to enhance the learning of wider representations with fewer parameters.

### 3.4. Evaluation Metrics

Because the model predicts numeric values, quantitative assessments of statistics are used as evaluation measurements. *R*-squared, which ranges from 0% to 100%, is used to show that the model is significantly better than the average total case value. To show the average error of the model on the corresponding days and to compare different forecasting models, root mean squared error (RMSE) and mean absolute error (MAE) metrics were used [15]. These metrics are commonly used to evaluate models and are typically applied to single time-series dataset. Equations (1)–(3) are the mathematical definitions of *R*-squared, RMSE, and MAE, respectively, where *y*_*i*_ is the *i*th observed value, ${\overset{⌢}{y}}_{i}$is the *i*th forecasted value, and *N* denotes the number of test data points. For qualitative assessments of statistics, visualizations of model outputs were formed to determine whether the models worked in certain areas.

(1) $$\begin{array}{c} R^{2}=1-\;\frac{\sum {\left(y_{i\;}–\;\overset{⌢}{y}\right)}^{2}}{\sum {\left(y_{i\;}–\;y^{\prime }\right)}^{2}}, \end{array}$$

(2) $$\begin{array}{c} \text{RMSE }=\;\sqrt{\frac{1}{N}\;\sum_{i=1}^{N}{\left(y_{i\;}–\;\overset{⌢}{y}\right)}^{2}}, \end{array}$$

(3) $$\begin{array}{c} \text{MAE }=\;\frac{1}{N}\;\sum_{i=1}^{N}{\left|y_{i\;}–\;\overset{⌢}{y}\right|}^{2}. \end{array}$$

## 4. Results and Discussion

The experiments were conducted on a Windows 10 ×64, Intel Core I i7-4770K CPU with 3.50 GHz and 16,0 GB DDR3 RAM. We implemented our experiment on the Keras framework in Python with the Jupiter Notebook. The hyperparameters selected for all models are shown in Table 2. The AdaBelief optimizer with learning rate scheduler warmup was selected because it adapts the step size based on the difference between predicted and observed gradients [34]. Additionally, gradient centralization was used as an optimization technique to improve convergence [33]. A threshold rectified linear unit (ReLU) flatten-T Swish was used as an activation function, with a threshold of −0.2, which allowed negative values to be propagated in the network and improved performance [35].

The past window parameter and the next parameter values were empirically selected. Enough training data were used to reduce the variance of the prediction to 0. Hence, 80% of the input data were selected for training. The algorithm was optimized by validating the model using a test dataset. The test data were collected from Saudi Arabian cases and then validated to evaluate the model efficiency. Thus, 20% was selected as the test data. The total number of parameters used was 2,933,993, including 2,933,941 trainable parameters and 52 nontrainable parameters. In total, we performed three (methods) × five (next values) = 15 experiments.

The prediction speeds of DNN, LSTM, and TM were 0.025, 0.016, and 0.036 s, respectively. The obtained models required an acceptable amount of computation time. This is because the ReLU layer reduced the complexity owing to a decrease in the training time. Nevertheless, the LSTM converged faster than the other models.

Each model was trained to predict the new cases instead of the overall cases to achieve a numerically stable model. Hence, to evaluate the model stability, the average total of new cases per batch was calculated according to the evaluation metrics, *R*-squared, RMSE, and MAE, over 1500–2000 epochs. Figures 7 and 8 show the *R*-squared and RMSE values of the average total new cases per batch, respectively. As can be seen from Figure 7, the TM achieved the highest values with training data but the lowest values with test data. Hence, TM was unstable with the test data. In contrast, as can be seen from Figure 8, the TM achieved the lowest values with training data but the highest values with test data. Hence, TM was unstable with the test data. Thus, it can be concluded that TM was overfitted and requires more data to perform better. However, the simpler models, DNN and LSTM, worked slightly better given the same data. Models continue training until they can classify the maximum testing data, which leads to high accuracy. It can be seen from Figures 7 and 8 that the amount of data was insufficient to train a robust model.

Figure 9 shows the prediction results of the three models. Each point in the predicted values is the number of cases per day, which is generated by using the observed number of cases from previous four days. Since the test dataset was used, the real day values for the forecasting were known. As can be seen from Figure 10, all models predicted values close to the real values. Thus, models were very accurate, and there is a strong correlation between all the model predictions and real values. All models have succeeded in predicting the total overall cases using the testing data.

After the models were trained, the overall RMSE values for DNN, LSTM, and TM were 1235.577, 241.933, and 526.3385, respectively. Additionally, the overall MAE values for DNN, LSTM, and TM were 931.2212, 166.332, and 362.7718, respectively. Finally, the overall MAE values for DNN, LSTM, and TM were 0.997, 0.999, and 0.999, respectively.

Table 3 shows the forecasting accuracy scores by day based on the evaluation metrics for each method for the next five days. The evaluation metrics were calculated based on the entire test on overall cases. The models predicted new cases and then added the values to the overall values. Hence, it is aggregated to new overall cases.

As previously stated, MAE is the absolute value of the difference between the forecasted and actual values; thus, the smaller the value, the better the model performance. The DNN had an error of approximately ±81 for the next day, which is better than that of the TM with an error of ±131. However, it dropped prediction to ±339 and ±431 for the 4th and 5th days ahead. This significant drop on later days indicates a poor forecasting ability. The LSTM model showed the best results for the testing data. It is clear from the table that LSTM can predict total overall cases for the new 85 days, which was not part of the training data, with an error of approximately ±66 cases for one day ahead. Then, it decreased to ±213 and ±273.

A small value of RMSE means that the values estimated by the model are close to the real values. LSTM has the highest accuracy based on the lowest RMSE obtained, followed by DNN and TM. As shown in Figure 10, the number of new cases in this interval ranges from ∼400 to ∼1300. Thus, LSTM exhibits the best performance among the three models.

Furthermore, the RMSE tends to be larger than MAE, especially when using TM, because the RMSE penalized significant errors more. Hence, more errors were detected, and the values of TM showed a larger error gap than those of the DNN and LSTM, with LSTM achieving better results. *R*-squared shows the proportion of the total variability by the model. The values of *R*-squared range from 0 to 1. In this case, all models achieved values of 1 or 0.99, which is within the accepted range of *R*-squared score. This indicates that the regression predictions perfectly fit the data.

## 5. Conclusion

This study addresses an important subject and introduces advanced technology in the field of infectious diseases. Moreover, it focuses on predicting disease transmission in Saudi Arabia and can be used by other countries affected by the disease. Analyzing and understanding the factors that increase the spread of COVID-19 in Saudi Arabia is essential to slowing the spread and preventing more infections. Investigating the link between the measures to combat the pandemic and disease spread will shed some light on the effectiveness of the applied preventive measures. This enables authorities to target their efforts for more effective actions.

In this study, we developed three prediction models using a DNN, LSTM, and transformer to show the influence of different factors on the transmission of SARS-CoV-2 in Saudi cities. The LSTM model obtained the best prediction results with a reasonable computation time. This model can help effectively control outbreaks and pandemics when new viruses emerge in the future.

In the future, we will consider more Saudi cities in the prediction model. Moreover, we intend to conduct a regression analysis to find the most influential factors impacting new cases. This study only used the following NN models: DNN, LSTM, and transformer. Future research should compare the performance of current models with convolutional neural networks and support vector machines on the same dataset.

## Figures and Tables

**Figure 1:** Status of COVID-19 in Saudi Arabia as of May 7, 2020.

**Figure 2:** Top 10 Saudi cities with the most COVID-19 cases as of May 7, 2020 [5].

**Figure 3:** Block diagram of the prediction model.

**Figure 4:** Total COVID-19 cases in Makkah Province.

**Figure 5:** The demographics of COVID-19 confirmed cases in Saudi Arabia as of May 7, 2020 [5].

**Figure 6:** Percentage change from baseline mobility data for Makkah Province from February 2020 to June 2021. (a) Retail and recreation. (b) Grocery and pharmacy. (c) Parks. (d) Transit stations. (e) Workplaces. (f) Residential.

**Figure 7:** Intermediate general stability values using *R*-squared average values for all models. (a) Training data using DNN. (b) Training data using LSTM. (c) Training data using TM. (d) Testing data using DNN. (e) Testing data using LSTM. (f) Testing data using TM.

**Figure 8:** Intermediate general stability values using RMSE average values for all models. (a) Training data using DNN. (b) Training data using LSTM. (c) Training data using TM. (d) Testing data using DNN. (e) Testing data using LSTM. (f) Testing data using TM.

**Figure 9:** Real versus predicted cases: maximum next predicted values using fully connected deep neural network (DNN), long short-term memory (LSTM), and transformer model (TM).

**Figure 10:** Number of new cases.

**Table 1:** Summary of data sources used for the study.

Data	Resource
Daily COVID-19 cases in Saudi Arabia	Ministry of Health—Dashboard of COVID-19 in Saudi [16]
Mobility data	Google COVID-19 Community Mobility Reports [3]

**Table 2:** Model hyperparameters.

Hyperparameter	Value
Optimizer	AdaBelief
Optimization technique	Gradient centralization (GC)
Activation function	FTS
Training data	80%
Test data	20%
Past window	30
Next values	5

**Table 3:** Forecasting accuracy using fully connected deep neural network (DNN), long short-term memory (LSTM), and transformer model (TM) methods for each predicted day.

	MAE					RMSE					*R* ^2^				
	Day 1	Day 2	Day 3	Day 4	Day 5	Day 1	Day 2	Day 3	Day 4	Day 5	Day 1	Day 2	Day 3	Day 4	Day 5
DNN	81.071	163.776	251.776	338.988	430.588	101.339	199.718	296.404	394.119	493.247	1.000	1.000	1.000	1.000	0.999
LSTM	66.153	117.188	162.753	212.506	273.059	86.619	158.978	222.056	286.454	358.490	1.000	1.000	1.000	1.000	1.000
Transformer	131.129	262.282	377.753	474.188	568.506	154.398	324.864	484.940	636.876	784.224	1.000	1.000	1.000	1.000	0.999

## Data Availability

The data used to support the findings of this study are included within the article and taken from the following websites: https://www.moh.gov.sa/en/Pages/default.aspx, 2020 and https://www.google.com/covid19/mobility/, 2020.
